RETRACTED

# Correlation Between Platelet-Lymphocyte Ratio and Neutrophil-Lymphocyte Ratio in Patients with Uterine Leiomyoma: A Cross-Sectional Study

**DOI:** 10.1155/2022/3257887

**Published:** 2022-08-11

**Authors:** Yanan Duan, Yiqing Peng, Xiuling Shi, Ying Zhao, Kunyan Liu, Runsheng Zhou, Cunxu Peng

**Affiliations:** ^1^Jining Medical University, Jining 272002, Shandong, China; ^2^Department of Gynecology, Affiliated Hospital of Jining Medical University, Jining 272029, Shandong, China

## Abstract

The inflammatory reaction has been proven to be a key factor in the pathogenesis of uterine leiomyoma. The platelet-lymphocyte ratio (PLR) and the neutrophil-lymphocyte ratio (NLR) are inexpensive and reliable inflammatory biomarkers. However, evidence of the relationship between PLR and NLR in patients with uterine leiomyoma is limited. This study aimed to explore the relationship between PLR and NLR in patients with incident uterine leiomyoma. This cross-sectional study included 763 patients with uterine leiomyoma who were first diagnosed in our hospital between January 2016 and December 2016. Patient characteristics were collected for univariate analysis, smooth curve fitting, and multivariate piecewise linear regression. Overall, 722 patients with an average age of 40.16 ± 5.99 years were included. The average PLR was 161.22 ± 65.33. Univariate analysis revealed a significant positive correlation between PLR and NLR (*P* < 0.0001). In addition, the non-linear relationship between the PLR and NLR was tested using smooth curve fitting after adjusting for potential confounding factors. The multivariate piecewise linear regression model showed that there was a significant positive correlation between PLR and NLR in both PLR <226.45 (*β* 0.01, 95% CI: 0.01, 0.01;*P* < 0.0001) and >226.45 (*β* 0.00, 95% CI: 0.00, 0.00; *P*=0.0026). In conclusion, PLR and NLR are positively correlated in patients with uterine leiomyoma. This result clarifies the promoting role of inflammation in the occurrence of uterine leiomyoma.

## 1. Introduction

Uterine leiomyoma (UL) is the most common benign uterine tumor among women of childbearing age. Its clinical symptoms include increased menstrual bleeding, dysmenorrhea, and infertility, which are some of the main causes of hysterectomy. [1–3] However, the pathogenesis of uterine leiomyoma remains unclear to date, although in-depth studies have shown that inflammatory reactions play an important role in the pathogenesis of the disease. [4, 5] A previous in vitro study [6] suggested that progenitor cells of uterine leiomyoma promote the development of uterine leiomyoma through the expression of related inflammatory factors. Current studies on uterine leiomyoma and inflammation [7, 8] focus on inflammatory factors such as interleukin-4 (IL-4), IL-5, IL-10, and IL-13, and evidence regarding the relationship between neutrophil-lymphocyte ratio (NLR) and platelet-lymphocyte ratio (PLR) in patients with uterine leiomyomas is limited.

RETRACTED

The NLR and PLR are easily accessible and replicable biological indicators of inflammation [9, 10]. The relationship between PLR and NLR has been widely studied in malignant tumors, cardio-cerebrovascular stroke, rheumatoid arthritis, and acute rheumatic fever, among other diseases. These two ratios can also indicate the occurrence and development of pre-eclampsia and eclampsia in pregnant women. In addition, they are related to the prognosis of gynecological tumors such as sarcoma and endometrial carcinoma. [11, 12] Recent literature [13, 14] has shown that PLR and NLR play an important role in distinguishing uterine leiomyoma from other diseases. This study aimed to clarify the relationship between PLR and NLR in patients with uterine leiomyoma to help further explain the role of inflammation in the occurrence and development of the disease.

## 2. Materials and Methods

### 2.1. Study Design and Population

This single-center cross-sectional study was approved by the Institutional Review Board of the Affiliated Hospital of Jining Medical University (approval number: 2022C114). Informed consent was not required owing to the traceability of the cohort study.

The subjects were patients diagnosed with uterine leiomyomas at the gynecology department of the Affiliated Hospital of Jining Medical University between January 2016 and December 2016. The inclusion criteria were as follows: (1) uterine leiomyoma diagnosed by auxiliary examination and preoperative clinical manifestation; (2) uterine leiomyoma diagnosed by postoperative pathology; and (3) diagnosis of uterine leiomyoma for the first time. The exclusion criteria were as follows: (1) treatment with antibiotics and antithrombotic drugs within 3 months preoperatively; (2) hematological diseases, malignant tumors, autoimmune diseases, metabolic diseases, hypersplenism, or existing infections; (3) treatment with glucocorticoids, permanent immunoregulatory drugs, or anti-inflammatory drugs; (4) age <18 years; (5) pregnant or lactating women; and (6) history of drug or surgical treatment for uterine leiomyoma.

The data, which did not include identifiable information to protect patient privacy, were obtained from the hospital's electronic medical record system. In total, 763 patients were initially evaluated.

### 2.2. Variables

Patients' data, including age, sex, body mass index (BMI), hypertension, heart disease, diabetes, and routine blood indices, were retrospectively collected. Routine blood indices were obtained during hospitalization as follows. After admission, peripheral venous blood was collected after an 8-hour fast and processed in the laboratory. All measurements were performed by laboratory technicians and inspectors in our hospital. PLR was calculated by dividing lymphocyte count by platelet count, and NLR was calculated as neutrophil count divided by lymphocyte count, using the same blood sample.

RETRACTED

### 2.3. Statistical Analysis

Normally distributed continuous variables were presented as the average ± standard deviation, while non-normally distributed continuous variables were presented as the median. Categorical variables were expressed as frequencies or percentages. The *χ*2 test, one-way analysis of variance, or Kruskal-Wallis test were used to compare differences in categorical variables, normally distributed variables, and nonnormally distributed variables among quartiles of NLR groups, respectively. Data analysis was divided into two steps. In step 1, multivariate linear regression models adjusted by patient characteristics and significant variables in the univariate analysis were created. In step 2, the generalized additive model and smooth curve fitting (punitive spline method) were conducted to address the nonlinear issues of NLR and PLR. If nonlinearity was detected, the recursive algorithm was first used to calculate the inflection point and then construct a two-piece linear regression on both sides of the inflection point. The optimal fitting model was determined based on the *P* value obtained from the logarithmic likelihood ratio test. A sensitivity analysis was performed to ensure the robustness of the data. We converted PLR to a categorical variable and calculated the *P* value of the trend to verify the results of NLR as a continuous variable and to observe the possibility of nonlinearity. All statistical analyses were performed using the *R* statistical package (https://www.R-project.org*R* Foundation) and EmpowerStats (https://www.empowerstats.com Journal X&Y Solutions, Inc., Boston, Massachusetts, USA). Statistical significance was set at a two-sided *P* value of <0.05.

## 3. Results

### 3.1. Baseline Patient Characteristics

In total, 722 participants were included in the final analysis (Figure 1). The baseline patient characteristics according to PLR quartiles are shown in Table 1. The average age of the patients was 40.16 ± 5.99 years. There were no significant differences in age, BMI, dysmenorrhea, the maximum diameter of myoma, hypertension, diabetes, heart disease, endometriosis, adenomyosis, adenomyoma, benign adnexal tumor, and neutrophil count among the PLR groups (all *P* > 0.05). Meanwhile, the regularity of menstruation, menstrual volume, and the number of leiomyomas were significantly different (all *P* < 0.05). Participants in the highest NLR quartile (Q4) had higher platelet counts, and NLR, and lower lymphocyte counts than those in the other quartile groups.

RETRACTED

### 3.2. Univariate Analysis of NLR

The results of univariate analysis are presented in Table 2. Univariate linear regression showed that age, BMI, menstrual regularity, dysmenorrhea, menstrual volume, and number of leiomyomas, maximum diameter of leiomyomas, hypertension, diabetes, heart disease, endometriosis, adenomyosis, adenomyoma, and benign adnexal tumors were not associated with NLR. Furthermore, univariate analysis showed that PLR was positively correlated with NLR (*β* 0.00, 95% CI: 0.00, 0.01).

### 3.3. Results of Adjusted Linear Regression

A model adjusted for confounding factors was built using multivariate linear regression to analyze the independent effect of PLR on NLR. The effect sizes (*β*) and 95% confidence intervals are listed in Table 3. In the unadjusted model (model 1), the size of the model-based effect could be interpreted as an increase of 1 unit in the PLR associated with NLR. For example, in the minimum adjustment model (model 2), when PLR increased by 1 unit, NLR increased by 0.01 unit (*β* 0.01, 95% CI: 0.01, 0.01). For the sensitivity analysis, PLR was converted from a continuous variable to a categorical variable (PLR quartile). In the minimum adjustment model and the fully adjusted model, the *P* value of the PLR trend was consistent with that when the PLR was a continuous variable.

Adjust II adjusts for: age, BMI, menstrual regularity, dysmenorrhea, menstrual volume, number of myomas, the maximum diameter of leiomyoma, hypertension, diabetes, heart disease, endometriosis, adenomyosis, adenomyoma, and benign adnexal tumors.

Adjust III adjusts for: age (smooth), BMI (smooth), menstrual regularity, dysmenorrhea, menstrual volume, number of myomas, the maximum diameter of leiomyoma (smooth), hypertension, diabetes, heart disease, endometriosis, adenomyosis, adenomyoma, and benign adnexal tumors.

### 3.4. Relationship between PLR and NLR

As shown in Figures 2(a) and 2(b), smooth curve fitting was performed after adjusting for possible confounding factors, including age, BMI, menstrual regularity, dysmenorrhea, menstrual volume, number of leiomyomas, the maximum diameter of leiomyoma, hypertension, diabetes, heart disease, endometriosis, adenomyosis, adenomyoma, and benign adnexal tumor. The NLR showed a non-linear relationship with PLR. Specifically, the NLR level increased as the PLR increased. As shown in Table 4, the threshold effects were further investigated based on the curve fitting. There was a significant positive correlation between PLR and NLR in both PLR <226.45 (*β* 0.01, 95% CI: 0.01, 0.01; *P* < 0.0001) and PLR >226.45 (*β* 0.00, 95% CI: 0.00, 0.00; *P*=0.0026).

RETRACTED

The LRT test and the logarithmic likelihood ratio test (*P* < 0.05 mean that model 2 is significantly different from model 1, which represents a nonlinear relationship).

Adjusted variables: age, BMI, menstrual regularity, dysmenorrhea, menstrual volume, number of leiomyomas, the maximum diameter of leiomyomas, hypertension, diabetes, heart disease, endometriosis, adenomyosis, adenomyoma, benign adnexal tumor. Statistical significance is set at*P* < 0.05.

There is an Independent correlation between PLR and NLR in patients with multiple uterine leiomyomas. A smooth fitting curve was drawn for patients with multiple uterine leiomyomas using the methods shown in Figures 2(a) and 2(b). In patients with multiple uterine leiomyomas, the NLR increased as the PLR increased (see Figure 3).

## 4. Discussion

The relationship between PLR and NLR has been widely studied in cancer, but this relationship is yet to be clarified in patients with uterine leiomyoma. The current study found a non-linear positive correlation between PLR and NLR in patients with uterine leiomyoma. Overall, the NLR increased as the PLR increased. Sensitivity and threshold effect analyses showed a significant positive correlation between PLR and NLR, which was also verified in patients with multiple uterine leiomyomas.

PLR, as indicative of the ratio of platelet counts to lymphocyte counts, can comprehensively present various inflammatory pathways associated with whole blood cells, and it has a higher predictive capability than platelet or lymphocyte count alone. [15] Several studies [16, 17] have indicated that PLR can be used as an indicator of cellular immune inflammation. In addition, PLR is an independent risk factor for the prognosis of coronavirus disease in 2019 [18, 19], and a high PLR is significantly associated with mortality. A clinical study [20] also showed that PLR is an independent risk factor for postoperative metastasis of malignant tumors, and a high PLR indicates a higher rate of postoperative metastasis. Several differential diagnosis studies [14, 21] have shown that PLR is an important index for establishing a predictive model for the diagnosis of leiomyoma. The NLR indicates the ratio of neutrophils to lymphocytes; importantly, it is an established index of inflammation and a prognostic index for many diseases [22]. Some studies [23] have shown that a higher NLR indicates poor overall survival in renal cell carcinoma. The NLR is also a reliable prognostic indicator for patients with various diseases and can be used as a biomarker of serum CA125 to diagnose endometriosis. [14].

RETRACTED

A study of uterine leiomyoma [24] has reported a significant difference in NLR between patients with uterine leiomyoma measuring >5 cm and those with tumors measuring <5 cm. A recent study [25] indicated that the NLR can be used to evaluate the inflammatory reaction of uterine leiomyoma. After activation, platelets release pro-inflammatory factors, such as recruiters and activators of leukocytes, and these participate in immune regulation and inflammatory function [26]. An animal study [27] showed that there is an obvious relationship between platelet count and leiomyoma, but the specific mechanism remains to be further studied. Neutrophil activation enhances the recruitment of many different cell types involved in acute and chronic inflammation, thus activating pro-inflammatory effects [28, 29]. A study in mice [30] showed a significant increase in the number of neutrophils and related cytokines in the peritoneal fluid of mouse models with endometriosis. For example, as one of the most common and inexpensive preoperative indicators, lymphocyte count is closely related to general health conditions and chronic inflammation [31]. A study [32] reported that a change in lymphocyte count is correlated with the release of pro-inflammatory mediators and infertility in uterine leiomyoma patients of childbearing age.

Uterine leiomyomas consist of smooth muscle and connective tissue, which may be linked to genetic factors, chromosomal abnormalities, and other factors. [2, 3] One study [33] concluded that various immune and tumor diseases are driven and maintained by inflammation in the early stage of uterine leiomyoma, and the abnormal inflammatory process perpetuates tissue damage, leading to chronic disease. Several studies [34–36] have pointed out that inflammation plays an important role in the pathogenesis of uterine leiomyoma, as well as in the development of fibroid fibrosis and disease progression. Many studies [20, 23, 37, 38] have also reported that PLR and NLR can reflect the inflammatory state of the body in the absence of infectious diseases. In the current study, NLR showed an upward trend with an increase in PLR in patients with multiple uterine fibroids. It was further clarified that the trends of PLR and NLR were consistent between single and multiple uterine leiomyomas.

The clinical value of this study is as follows: (1) to the best of our knowledge, this is the first study to investigate the independent association between NLR and PLR in patients newly diagnosed with uterine leiomyoma. (2) the relationship between NLR and PLR may help further explain the role of inflammation in the occurrence and development of uterine leiomyoma. (3) our study findings can widen the role of NLR and PLR as markers of inflammation in various diseases. However, this study also had some limitations. First, the subjects included were newly diagnosed with uterine leiomyomas. Thus, the findings may have limited generalizability. In addition, the dynamic variation in NLR and PLR was not investigated because of inevitable selection and evaluation biases. Given the exclusion criteria, the findings cannot be extended to the population of patients with hematological diseases, other malignant tumors, autoimmune diseases, metabolic diseases, or existing infections; patients treated with glucocorticoids, permanent immunomodulatory, or anti-inflammatory drugs; or those aged <18 years. These populations should be considered in future studies.

RETRACTED

## 5. Conclusions

In conclusion, PLR and NLR are positively correlated in patients with uterine leiomyoma. This result clarifies the promoting role of inflammation in the occurrence of uterine leiomyoma.

## Figures and Tables

**Figure 1:** Patient inclusion flowchart.

**Figure 2:** Relationship between PLR and NLR. (a) The smooth fitting curve of PLR and NLR. (b) The scatter diagram for PLR and NLR distributions. The solid red line denotes a smooth curve fitting between the variables. The blue band denotes the 95% confidence interval for the fit. The model is adjusted for age, BMI, menstrual regularity, dysmenorrhea, menstrual volume, the maximum diameter of leiomyoma, hypertension, diabetes, heart disease, endometriosis, adenomyosis, adenomyoma, and benign adnexal tumor.

**Figure 3:** Relationship between PLR and NLR in patients with multiple uterine leiomyomas. (a) The smooth fitting curve of PLR and NLR. (b) The scatter diagram of PLR and NLR distributions. The solid red line denotes a smooth curve fitting between the variables. The blue band denotes the 95% confidence interval for the fit. The model is adjusted for age, BMI, menstrual regularity, dysmenorrhea, and menstrual volume, the maximum diameter of leiomyoma, hypertension, diabetes, heart disease, endometriosis, adenomyosis, adenomyoma, and benign adnexal tumor.

**Table 1:** Baseline patient characteristics by PLR quartile.

Characteristic	PLR (min–max)				
	Q1 (50.82–117.9)	Q2 (118–145.9)	Q3 (146.3–190.9)	Q4 (191–662.6)	*P* value
*N*	182	177	180	183	
Age (years, mean ± SD)	39.90 ± 6.66	40.13 ± 6.14	39.89 ± 5.40	40.72 ± 5.70	0.518
BMI (kg/m^2^, mean ± SD)	24.55 ± 3.25	24.66 ± 3.32	24.50 ± 3.20	24.04 ± 2.99	0.266
Menstrual regularity, *n* (%)					0.043
Regular	179 (98.35)	173 (97.74)	178 (98.89)	173 (94.54)	
Irregular	3 (1.65)	4 (2.26)	2 (1.11)	10 (5.46)	
Dysmenorrhea, *n* (%)					0.576
No	141 (77.47)	142 (80.23)	138 (76.67)	150 (81.97)	
Yes	41 (22.53)	35 (19.77)	42 (23.33)	33 (18.03)	
Menstrual volume					0.026
Low	10 (5.49)	6 (3.39)	8 (4.44)	3 (1.64)	
Moderate	155 (85.16)	146 (82.49)	149 (82.78)	141 (77.05)	
High	17 (9.34)	25 (14.12)	23 (12.78)	39 (21.31)	
Number of myomas					0.014
Single	113 (62.09)	112 (63.28)	92 (51.11)	92 (50.27)	
Multiple	69 (37.91)	65 (36.72)	88 (48.89)	91 (49.73)	
Maximum diameter of myoma (cm)	5.62 ± 2.55	5.90 ± 2.43	5.57 ± 2.31	6.05 ± 2.31	0.188
Hypertension, *n* (%)					0.727
No	180 (98.90)	174 (98.31)	177 (98.33)	182 (99.45)	
Yes	2 (1.10)	3 (1.69)	3 (1.67)	1 (0.55)	
Diabetes, *n* (%)					0.555
No	181 (99.45)	175 (98.87)	179 (99.44)	183 (100.00)	
Yes	1 (0.55)	2 (1.13)	1 (0.56)	0 (0.00)	
Heart disease, *n* (%)					0.285
No	182 (100.00)	175 (98.87)	179 (99.44)	183 (100.00)	
Yes	0 (0.00)	2 (1.13)	1 (0.56)	0 (0.00)	
Endometriosis, *n* (%)					0.809
No	171 (93.96)	169 (95.48)	173 (96.11)	174 (95.08)	
Yes	11 (6.04)	8 (4.52)	7 (3.89)	9 (4.92)	
Adenomyosis and adenomyoma, *n* (%)					0.700
No	176 (96.70)	170 (96.05)	176 (97.78)	179 (97.81)	
Yes	6 (3.30)	7 (3.95)	4 (2.22)	4 (2.19)	
Benign adnexal tumor, *n* (%)					0.361
No	109 (59.89)	113 (63.84)	115 (63.89)	126 (68.85)	
Yes	73 (40.11)	64 (36.16)	65 (36.11)	57 (31.15)	
Platelet count (10^9^/L, mean ± SD)	225.96 ± 44.86	261.44 ± 50.13	286.46 ± 59.92	355.84 ± 84.00	<0.001
Neutrophil count (10^9^/L, mean ± SD)	3.32 ± 1.11	3.18 ± 1.17	3.04 ± 0.98	3.25 ± 1.23	0.107
Lymphocyte count (10^9^/L, mean ± SD)	2.34 ± 0.51	2.00 ± 0.38	1.74 ± 0.38	1.46 ± 0.34	<0.001
NLR (mean ± SD)	1.46 ± 0.51	1.61 ± 0.53	1.81 ± 0.67	2.28 ± 0.84	<0.001
PLR (mean ± SD)	97.68 ± 13.77	131.11 ± 8.30	165.52 ± 12.86	249.32 ± 61.22	<0.001

RETRACTED

**Table 2:** Univariate analysis of NLR.

Covariate	Statistics	*β* (95% CI)	*P*-value
Age (years)	40.16 ± 5.99	−0.00 (−0.01, 0.01)	0.5207
BMI (kg/m^2^)	24.43 ± 3.19	0.01 (−0.01, 0.02)	0.3456
Menstrual regularity, *n* (%)			
Regular	703 (97.37)	Reference	
Irregular	19 (2.63)	0.13 (−0.20, 0.46)	0.4436
Dysmenorrhea *n* (%)			
No	571 (79.09)	Reference	
Yes	151 (20.91)	−0.10 (−0.23, 0.02)	0.1137
Menstrual volume			
Low	27 (3.74)	Reference	
Moderate	591 (81.86)	0.31 (0.03, 0.58)	0.0312
High	104 (14.40)	0.19 (-0.11, 0.50)	0.2165
Number of myomas			
Single	409 (56.65)	Reference	
Multiple	313 (43.35)	0.09 (−0.01, 0.20)	0.0810
Maximum diameter of myoma (cm)	5.79 ± 2.40	0.02 (−0.01, 0.04)	0.1670
Hypertension *n* (%)			
No	713 (98.75)	Reference	
Yes	9 (1.25)	−0.26 (−0.74, 0.21)	0.2768
Diabetes *n* (%)			
No	718 (99.45)	Reference	
Yes	4 (0.55)	0.06 (−0.65, 0.77)	0.8685
Heart disease *n* (%)			
No	719 (99.58)	Reference	
Yes	3 (0.42)	−0.15 (−0.97, 0.67)	0.7168
Endometriosis			
No	687 (95.15)	Reference	
Yes	35 (4.85)	0.08 (−0.16, 0.33)	0.5177
Adenomyosis, adenomyoma			
No	701 (97.09)	Reference	
Yes	21 (2.91)	0.07 (−0.24, 0.38)	0.6579
Benign adnexal tumor			
No	463 (64.13)	Reference	
Yes	259 (35.87)	−0.05 (−0.16, 0.06)	0.3776
PLR (mean ± SD)	161.22 ± 65.33	0.00 (0.00, 0.01)	<0.0001

**Table 3:** Relationship between PLR and NLR in different models.

Variable	Unadjusted model I		Adjusted model II		Adjusted model III	
	*β* (95% CI)	*P* value	*β* (95% CI)	*P* value	*β* (95% CI)	*P* value
PLR	0.00 (0.00, 0.01)	<0.0001	0.01 (0.00, 0.01)	<0.0001	0.00 (0.00, 0.01)	<0.0001
PLR (quartile)						
Q1 (50.82–117.9)	Reference		Reference		Reference	
Q2 (118–145.9)	0.15 (0.01, 0.28)	0.0343	0.15 (0.01, 0.29)	0.0316	0.14 (0.00, 0.28)	0.0434
Q3 (146.3–190.9)	0.35 (0.21, 0.48)	<0.0001	0.36 (0.22, 0.49)	<0.0001	0.34 (0.21, 0.48)	<0.0001
Q4 (191–662.6)	0.81 (0.68, 0.95)	<0.0001	0.84 (0.71, 0.98)	<0.0001	0.83 (0.70, 0.97)	<0.0001

**Table 4:** Threshold effect analysis of the relationship between PLR and NLR levels.

	NLR	
	Adjusted *β* value (95% CI)	*P* value
Model I		
One linear effect	0.00 (0.00, 0.01)	<0.0001
Model II		
Break point (*k*)	226.45	
<226.45 segment effect 1	0.01 (0.01, 0.01)	<0.0001
>226.45 segment effect 2	0.00 (0.00, 0.00)	0.0026
Effect difference between 2 and 1	−0.00 (−0.01, −0.00)	0.0017
Predicted value of equation at break point	2.24 (2.14, 2.34)	
LRT test		0.001

Model 1: Linear analysis, Model 2: Nonlinear analysis.

## Data Availability

The data used to support the findings of this study has been included in this article.
